# Factors Affecting the Self-Isolation Monitoring Program for COVID-19 Patients at the Universitas Indonesia Hospital

**DOI:** 10.1155/2022/2297328

**Published:** 2022-08-24

**Authors:** Rakhmad Hidayat, Zlatikha Djuliannisaa, Alyssa Putri Mustika, Gemia Clarisa Fathi, Muhammad Hafiz Aini, Wahyu Ika Wardani, Assifa Swasti Anindita, Siti Azizah, Astuti Giantini, Muhammad Arza Putra

**Affiliations:** ^1^Faculty of Medicine, Universitas Indonesia, Jakarta, Indonesia; ^2^Cipto Mangunkusumo Hospital, Jakarta, Indonesia; ^3^Universitas Indonesia Hospital, Depok, Indonesia

## Abstract

When the outbreak of the COVID-19 delta variant occurred in June 2021, there was a marked increase in Indonesia's number of self-isolated patients. The Universitas Indonesia Hospital provided a One-Stop Service (OSS) to monitor COVID-19 patients on self-isolation. This study was conducted to determine the effectiveness of the self-isolation monitoring performed by hospitals and the factors that determined the outcomes of patients on self-isolation. This study was conducted using a cross-sectional method based on secondary data from electronic medical records. Data analysis was performed by determining the relationship of patient risk factors and characteristics with COVID-19 outcomes. The study found that poorer symptoms, administration of antibiotics, absence of shortness of breath, and normal ALT levels significantly improved the outcome of OSS patients. The study also suggested that during monitoring of patients on COVID-19 self-isolation, chest/thorax radiography is necessary. The self-isolation monitoring program is essential to observe the patient's condition and evaluate the possibility of deteriorating conditions that could lead to admission decisions in the early or middle stages of the program. This will be beneficial during pandemic emergencies.

## 1. Introduction

From June 28, 2021, to July 30, 2021, the number of confirmed cases of COVID-19 in Indonesia experienced a twofold increase, with the number of deaths increasing by nearly 50%. [1] This occurred during the delta variant outbreak, and based on government data, the delta variant comprised 98.9% of COVID-19 cases. [2] At this time, there was a notable increase in the rate of emergencies and utilization of hospital resources. Data from a hospital in Indonesia noted that there were 63 deaths in one day, and 33 deaths occurred once the central oxygen supply was exhausted. According to the Indonesian Doctors Association, more than 400 doctors have died in Indonesia since the pandemic started. [3] The number of cases in Jakarta increased by 35% during this period, with the highest number of patients on self-isolation reaching 88,295. [4, 5] Accordingly, many people were infected with COVID-19 and underwent self-isolation. This required attention and supervision from health workers at the hospital in order to achieve effective self-isolation.

Under supervision, health workers must assess a patient's overall condition. To optimize observation and prevent patient deterioration, the symptoms, physical examination, and support that can affect the outcome of COVID-19 patients must be known. Thus, immediate treatment can be performed on patients with deterioration, given that the bed occupancy rate in Jakarta once reached 100%, which made it challenging for patients with deteriorating conditions to receive hospital treatment. [6–8] A similar incident also occurred in Singapore, where 89% of hospital beds for isolation patients were occupied, and patients requiring further treatment experienced difficulties. [9] Therefore, this study was conducted to identify factors that affected the outcomes of patients on COVID-19 self-isolation.

The Universitas Indonesia Hospital created an independent isolation monitoring program (One Stop Service (OSS)), where patients came in private vehicles and underwent symptom assessment, vital sign evaluation, blood tests, thoracic radiography, drug administration, and monitoring of the patient's clinical condition over two weeks. This study was conducted to determine the effectiveness of the self-isolation monitoring performed by hospitals and the factors that affected the deterioration of patients on self-isolation.

## 2. Materials and Methods

This cross-sectional study used secondary data (from the electronic medical records) of patients who participated in the Universitas Indonesia Hospital self-isolation observation program from June 28, 2021, to July 30, 2021. The study included patients on COVID-19 self-isolation. At this stage, there were 206 patients. We excluded COVID-19 patients who were lost to follow-up or did not complete the self-isolation program, which finally resulted in 197 patients. Data collection consisted of the patient's symptoms, physical examination, laboratory findings, radiology results, and patient outcomes. The data were analyzed by evaluating the association between the risk factors and the effects of the self-isolation monitoring program. Descriptive statistics were used in the study. The chi-squared test was used to determine the direct effect of risk factors, with patient outcomes as the dependent variable. We use SPSS 26 for the statistic process, and we consider significant result if *p*-value <0.05.

This research was approved by The Ethics Committee of Universitas Indonesia Hospital, approval number S-009/KETLIT/RSUI/II/2022 with protocol number 2021-09-098. This research also followed the Declaration of Helsinki guidelines. The Ethics Committee of Universitas Indonesia Hospital granted a waiver of informed consent due to retrospective data collection, and guaranteed the privacy of the participant in this research was maintained with confidentiality.

## 3. Results

There were more female patients (56.35%) than male patients (43.65%) (Table 1) among the 197 patients. Most patients were over 45 years of age (48.73%). More patients were clinically asymptomatic or mildly symptomatic (65.48%) than moderately or severely symptomatic (34.51%).

The patients' characteristics are presented in Table 2 and included sex, age <45 years and >45 years, and the clinical severity of the COVID-19 disease. The patients were also divided into asymptomatic patients and those with mild, moderate, and severe symptoms. The patients were also monitored to determine whether they had completed the OSS follow-up program conducted by the Universitas Indonesia Hospital. We assessed the administration of antivirals and antibiotics and the history of vaccination before the patient was infected with COVID-19. The degree of symptom severity significantly affected patient outcomes. The use of antibiotics also significantly increased the risk of unimproved patient outcomes (*p* < 0.005).

Twelve main symptoms were assessed in patients undergoing COVID-19 self-isolation, including fever, cough, runny nose, shortness of breath, fatigue, myalgia, anosmia, headache, sore throat, nausea and vomiting, diarrhea, and ageusia (Table 3). Shortness of breath had the most significant effect on outcomes among the patients (*p*=0.001).

Table 4 shows several laboratory tests performed on the patients as part of the Universitas Indonesia Hospital self-isolation monitoring program, including C-reactive protein (CRP), erythrocyte sedimentation rate, alanine aminotransferase (ALT), hemoglobin, hematocrit, and neutrophil-lymphocyte ratio (NLR). However, some patients did not undergo these examinations, and were included in another category. The analysis found that a normal ALT level was a significant predictor of improved COVID-19 outcomes among self-isolated patients (*p* < 0.05).

Table 5 shows the results of the radiological examinations. The patients were divided into several categories based on the presence of abnormalities in the thoracic radiography results. Radiological test results were not significant determinants of outcomes among patients undergoing COVID-19 self-isolation. No significant trend showed that patients without abnormalities had a better improvement.

Table 6 shows that physical examinations were performed when the patient first visited to participate in the self-isolation program. Examinations included blood pressure, oxygen saturation, temperature, and pulse. However, some patients did not come in person; therefore, some examination data could not be obtained, and they were excluded from the total sample for this category. The data were not well distributed among all physical examinations; therefore, no significant parameter was found to determine patient outcomes. However, patients who had poor initial saturation had the 3.403-fold potential to experience deterioration. A crucial physical examination, chest auscultation, was difficult to perform using the drive-thru method.

## 4. Discussion

### 4.1. Patient Characteristics

The degrees of mild, moderate, and severe COVID-19 are distinguished by the presence of shortness-of-breath symptoms and desaturation, which indicate pneumonia in the patient. [10] A study by Kim et al. of young COVID-19 patients showed that mild or asymptomatic disease was associated with more stable manifestations. In contrast, patients with symptoms had a greater risk of pneumonia or deteriorating computerized tomography (CT) results. [11] This was supported by Shi et al., who reported a significant difference between patients with and without pneumonia in terms of improvement rates. [12] Both studies aligned with the current study, where patients with mild or asymptomatic COVID-19 had a 6.5-fold higher possibility of improved outcomes compared to patients with moderate and severe symptoms (*p* < 0.001).

The proportion of COVID-19 patients with secondary bacterial coinfections was 6.9%, based on the study by Langford et al. [13] Chedid et al. also reported that the average duration of secondary infections was 17 days in the non-survivor group and 14 days in the survivor group. [14] Therefore, Sieswerda et al. recommended empiric antibiotics for COVID-19 patients who were treated and had undergone bacterial culture. [15] In the current study, the use of antibiotics was significantly associated with unimproved patient outcomes. This is in contrast with the function of antibiotics, which helped overcome the secondary infections in COVID-19. The possibility is that in the current study, antibiotics were administered more often to patients with moderate-to-severe COVID-19 symptoms, showing a significant relationship with deterioration.

However, in a study conducted by Tanioka et al., the use of penicillin antibiotics was positively associated with mortality in COVID-19 patients. In contrast, other antibiotics such as cephalosporins, macrolides, and quinolones prevented mortality, although not significantly. [16] Thus, it cannot be ruled out that some antibiotics increase the likelihood of adverse outcomes in COVID-19 patients.

### 4.2. Clinical Manifestations

This study found that shortness of breath was a vital predictor of outcomes in COVID-19 patients, who were categorized based on severity, starting from improvement to death. [4, 5] The findings aligned with those of a systematic review and meta-analysis conducted by Shi et al., in which shortness of breath had a positive relationship with mortality outcomes in COVID-19 patients, while other significant symptoms did not demonstrate any significant associations. [12] Yang et al. also reported a significant association between dyspnea and mortality risk (odds ratio (OR): 4.52, 95% CI: 3.15–6.48, *p* < 0.001). [17] This was in line with the findings of the current study, in which patients who did not have shortness of breath as the major symptom had a reduced rate of deterioration, including lower mortality, than patients with shortness of breath.

In this study, fever, cough, headache, nausea, and vomiting showed no significant relationship with COVID-19 outcomes. This result was supported by a study conducted by Yang et al. Another symptom of COVID-19, fatigue, showed a significant association in their study (OR: 4.52, 95% CI: 3.15–6.48, *p* < 0.001), while this study found no significant association. [17].

### 4.3. Physical Examination

In the supervision of COVID-19 self-isolation patients, an initial physical examination was performed to determine the patient's primary condition and degree of illness. The tests included blood pressure, temperature, oxygen saturation, pulse rate, and respiratory rate. Oxygen saturation was found in all physical examinations to significantly predict the outcome of patients undergoing COVID-19 self-isolation. Based on studies by Mejia et al. and Xie et al., saturation below 90% or desaturation strongly predicted mortality in COVID-19 patients. [18, 19] Although no studies have revealed that normal oxygen saturation is a determinant of a good prognosis in COVID-19 patients, low oxygen saturation is closely related to deterioration. This study found that patients with normal oxygen saturation could achieve a 3.4-fold higher improvement in outcomes compared to hypoxemic patients. A larger number of samples is needed to obtain statistically significant results. [10, 11].

### 4.4. Radiological Examination

Thoracic radiological examination is usually mandatory in COVID-19 patients where pulmonary consolidation that leads to pneumonia can be found. Cozzi et al. divided chest radiology findings based on the zone of consolidation into peripheral, lower, unilateral, and bilateral zones. [20] The study also divided the severity of the thoracic radiology findings based on the zoning system, which included only one lobe, more than one lobe, and bilateral consolidation. In their study, chest radiography had a sensitivity of 68.1% and was related to the risk of ICU admission or outcomes in COVID-19 patients. [20] Mushtaq et al. and Toussie et al. employed a scoring system to determine the severity of chest radiograph findings. Both studies showed that the severity of the initial thoracic findings was a significant determinant of outcomes among patients with COVID-19. [21, 22] The current study found that, compared to those with abnormal radiographs, patients with normal thoracic radiographs had a 3.5-fold higher chance of improved COVID-19 outcomes. The less significant result noted in this study was possibly due to the fact that radiological abnormalities were not divided more precisely. In contrast, the more severe the radiological abnormalities, the worse the prognosis.

### 4.5. Laboratory and Outcome Predictors

This study found no significant association between the outcomes of COVID-19 patients and CRP level. This result differed from those of Ahnach et al. and Luo et al., who found that CRP was an independent risk factor for COVID-19. [23,24] Luo et al. also showed that CRP level had a good sensitivity of 90.5% and specificity of 77.6%. [24] Although the current study did not find a significant association, the proportion of patients with elevated CRP levels was relatively high (62%). This result supports the findings of Chen et al. and Zhang et al., who reported that elevated CRP levels occurred in 93% and 91% of patients, respectively. [25, 26].

A study by Leulseged et al. showed no significant association between COVID-19 severity and hematocrit levels. [27] Their results were in line with that of our study, which found no significant association between these two parameters.

Some studies have found that NLR is a predictor of COVID-19 outcomes. Yang et al. concluded that NLR was an independent factor in COVID-19 outcome (HR 2.46, 95% CI: 1.98–4.57). [28] A study by Lagunas and Rangel also found a significant association between these variables. [29] The current study showed different results, as only 12.5% of patients with an elevated NLR had poor outcomes.

This study found that ALT levels determined the outcome in COVID-19 patients. This is due to impaired liver function in COVID-19 patients. Kumar et al. found that ALT levels were elevated in COVID-19 patients. The relative risk for abnormal ALT levels was also higher in patients with severe COVID-19. [30] High liver enzyme levels were also found in COVID-19 patients with a significantly normal liver enzyme baseline in the study by Gholizadeh et al. [31] These two studies suggested that an increase in ALT levels was indirectly associated with COVID-19, especially in the more severe disease. Few studies have directly reported the association between elevated liver enzymes and COVID-19 outcomes or severity. However, the study revealed that lower ALT liver enzyme levels significantly affected the outcomes in COVID-19 patients on self-isolation. Further research is needed to determine the pathophysiology and the mechanism of liver damage in patients with COVID-19, which causes high levels of these liver enzymes. [11–13].

## 5. Conclusion

A major COVID-19 symptom, namely shortness of breath, significantly influenced the outcome of COVID-19 patients on self-isolation. Routine serum ALT assessment is recommended in these patients because ALT is a significant predictor of COVID-19 outcomes. The study strongly suggests that if a patient experienced shortness of breath, self-isolation should not be performed. Since there was a high chance of a worse outcome, our findings should improve the quality of service and monitoring of COVID-19 self-isolation patients to provide better results. This study was limited by the small number of samples compared to the total number of patients nationally and by the narrow time interval of data collection.

## Figures and Tables

**Table 1:** Demography of COVID-19 self-isolation patients.

	Frequency (percentage)
Gender	
Male	86 (43.65%)
Female	111 (56.35%)

Age	
18–45 years old	89 (45.18%)
<18 years old	12 (6.09%)
>45 years old	96 (48.73%)

Clinical degree	
Asymptomatic-mild	129 (65.48%)
Moderate-severe	68 (34.51%)

Antiviral	
Yes	124 (62.95%)
No	73 (37.05%)

Antibiotic	
Yes	136 (69.04%)
No	61 (30.96%)

**Table 2:** Clinical data of COVID-19 self-isolation patients.

	Outcome		*p* value	OR	CI
	Better	Worse			
Gender					
Male	102 (51.8%)	9 (4.6%)	0.994^*∗*^	1.004	0.358–2.814
Female	79 (40.1%)	7 (3.6%)			

Age					
<45 years old	96 (48.7%)	5 (2.5%)	0.095^*∗*^	2.485	0.830–7.440
>45 years old	85 (43.1%)	11 (5.6%)			

Clinical degree					
Asymptomatic-mild	124 (62.9%)	4 (2.0%)	0.000^*∗*^	6.526	2.017–21.117
Moderate-severe	57 (28.9%)	12 (6.1%)			

Vaccine					
Yes	132 (67.0%)	13 (6.6%)	0.469^*∗*^	0.622	0.170–2.275
No	49 (24.9%)	3 (1.5%)			

Antiviral					
Yes	111 (56.3%)	13 (6.6%)	0.114^*∗*^	0.366	0.101–1.330
No	70 (35.5%)	3 (1.5%)			

Antibiotic					
Yes	123 (62.4%)	15 (7.6%)	0.031^*∗*^	0.141	0.018–1.096
No	58 (29.4%)	1 (0.5%)			

*∗*Chi-square.

**Table 3:** Main symptoms and outcomes of COVID-19 self-isolation patients.

	Outcome		*p* value	OR	CI
	Better	Worse			
Fever					
Yes	78 (39.60%)	8 (4.10%)	0.593^*∗*^	0.757	0.272–2.107
No	103 (52.30%)	8 (4.10%)			

Cough					
Yes	146 (74.10%)	15 (7.60%)	0.194^*∗*^	0.278	0.036–2.177
No	35 (17.80%)	1 (0.50%)			

Runny nose					
Yes	54 (27.40%)	4 (2.00%)	0.684^*∗*^	1.276	0.394–4.133
No	127 (64.50%)	12 (6.10%)			

Shortness of breath					
Yes	22 (11.20%)	7 (3.60%)	0.001^*∗*^	0.178	0.060–0.526
No	159 (80.70%)	9 (4.60%)			

Fatigue					
Yes	8 (4.10%)	2 (1.00%)	0.158^*∗*^	0.324	0.063–1.673
No	173 (87.80%)	14 (7.10%)			

Anosmia					
Yes	65 (33.00%)	4 (2.00%)	0.38^*∗*^	1.681	0.521–5.425
No	116 (58.90%)	12 (6.10%)			

Headache					
Yes	45 (22.80%)	2 (1.00%)	0.266^*∗*^	2.316	0.507–10.584
No	136 (69.00%)	14 (7.10%)			

Sore throat					
Yes	13 (6.60%)	1 (0.50%)	0.889^*∗*^	1.161	0.142–9.492
No	168 (85.30%)	15 (7.60%)			

Nausea and vomiting					
Yes	39 (19.80%)	6 (3.00%)	0.145^*∗*^	0.458	0.157–1.338
No	142 (72.10%)	10 (5.10%)			

Diarrhoea					
Yes	24 (12.20%)	2 (1.00%)	0.931^*∗*^	1.07	0.229–5.004
No	157 (79.70%)	14 (7.10%)			

Ageusia					
Yes	15 (7.60%)	2 (1.00%)	0.565^*∗*^	0.633	0.131–3.050
No	166 (84.30%)	14 (7.10%)			

^*∗*^Chi-square.

**Table 4:** Laboratory results and outcomes of COVID-19 self-isolation patients.

	Outcome		*p* value	OR	CI
	Better	Worse			
CRP					
Normal	69 (35.60%)	4 (2.10%)	0.362*∗*	1.752	0.528–5.632
Increasing	110 (56.70%)	11 (5.70%)			

SGPT					
Normal	148 (76.30%)	9 (4.60%)	0.032*∗*	3.183	1.056–9.525
Increasing	31 (16.00%)	6 (3.10%)			

ESR					
Normal	51 (26.20%)	2 (1.00%)	0.21*∗*	2.57	0.560–11.792
Increasing	129 (66.20%)	13 (6.70%)			

Hb					
Normal	169 (87.10%)	13 (6.70%)	0.232*∗*	2.6	0.515–13.133
Anaemia	10 (5.20%)	2 (1.00%)			

Haematocrit					
Normal	164 (84.50%)	14 (7.20%)	0.817*∗*	0.781	0.096–6.355
Increasing	15 (7.70%)	1 (0.50%)			

NLR					
Normal	151 (77.80%)	11 (5.70%)	0.269*∗*	1.961	0.583–6.598
Increasing	28 (14.40%)	4 (2.10%)			

CRP: C-reactive protein; ESR: Erythrocyte sedimentation rate; ALT: Alanine aminotransferase; Hb: Hemoglobin; NLR: Neutrophil-lymphocyte ratio. *∗*Chi-square.

**Table 5:** Radiology results and outcomes of self-isolated COVID-19 patients.

	Outcome		*p* value	OR	CI
	Better	Worse			
Chest X-ray					
Normal	63 (32.60%)	2 (1.00%)	0.083*∗*	3.561	0.779–16.282
Abnormalities	115 (59.60%)	13 (6.70%)			

*∗*Chi-square.

**Table 6:** Physical examinations and outcomes of COVID-19 self-isolation patients.

	Outcome		*p* value	OR	CI
	Better	Worse			
Temperature					
Normal	138 (83.60%)	15 (9.10%)	0.868	0.836	0.101–6.935
Fever	11 (6.70%)	1 (0.60%)			

Blood pressure					
Normal	101 (58.40%)	11 (6.40%)	0.259	0.474	0.127–1.772
Hypertension	58 (33.50%)	3 (1.70%)			

Pulse					
Normal	120 (67.80%)	13 (7.30%)	0.28	0.441	0.245–1.934
Tachycardia	42 (23.70%)	2 (1.10%)			

Saturation					
Normal	35 (18.00%)	1 (0.50%)	0.218	3.403	0.433–26.754
Hypoxia	144 (74.20%)	14 (7.20%)			

*∗*Chi-square.

## Data Availability

The datasets generated and/or analyzed during the current study are not publicly available due to patients' privacy concerns but are available from the corresponding author on reasonable request.
